The article "Clinical Efficacy and Safety Analysis of Levofloxacin for the Prevention of Infection after Traumatic Osteoarthrosis and Internal Fixation: Systematic Review and Meta-Analysis" was retracted in 2023. Reasons: signs of a paper mill; compromised peer review; unreliable results or conclusions.

# Clinical Efficacy and Safety Analysis of Levofloxacin for the Prevention of Infection after Traumatic Osteoarthrosis and Internal Fixation: Systematic Review and Meta-Analysis

**DOI:** 10.1155/2022/8788365

**Published:** 2022-09-29

**Authors:** Weiliang Wang, ChuanQi Zou, Jie Zhang

**Affiliations:** ^1^Department of Traumatology, Beijing Daxing District People's Hospital, Beijing 102600, China; ^2^Department of Orthopedics, Banan Hospital of Chongqing Medical University, Chongqing 400000, China; ^3^Department of Pharmacy, The First Affiliated Hospital of Nanchang University, Nanchang, Jiangxi 330001, China

## Abstract

**Objective:**

Levofloxacin has been widely used in clinical anti-infection treatment; however, its adverse reactions to levofloxacin were also obvious in patients. Herein we aimed to systematically evaluate the clinical efficacy and safety of systemic administration of levofloxacin in the prevention of postoperative infection after traumatic osteoarthrosis and internal fixation.

**Methods:**

PubMed, Cochrane Library, OVID, EBSCO, CNKI, VIP database, and Wanfang Database were searched from December 1993 to December 2021. Meanwhile, China ADR Information Bulletin and WHO Pharmaceutical were searched manually. Newsletter and FDA Drug Safety Newsletter, also to retrieve the Websites of Chinese, Chinese, and drug regulatory authorities; To obtain data on adverse events in children with systemic administration of levofloxacin. The literature was screened according to inclusion and exclusion criteria. The risk of bias was evaluated for the included RCT literature.

**Results:**

There was a statistical difference in the comparison of the incidence of fever between the experimental group and the control group (OR = 2.29, 95% CI (1.75,2.98),*P* < 0.00001, I^2^ = 0%, *Z* = 6.11); elevated white blood cell count (OR = 1.82, 95% CI (1.31,2.52),*P*=0.0003, I^2^ = 0%, *Z* = 3.60); incidence of wound infection (OR = 2.11, 95% CI (1.54,2.90),*P* < 0.00001, I^2^ = 0%, *Z* = 4.64); adverse drug reaction (OR = 1.82, 95% CI (1.21,2.74),*P*=0.004, I^2^ = 0%, *Z* = 2.86).

**Conclusion:**

In the clinical use of levofloxacin, adverse drug reactions including fever, elevated white blood cell count, and wound infection should be concerned.

## 1. Introduction

With the development of modern medical science, the types of orthopedic trauma treatment and internal fixation are also increasing, and actively dealing with the prognosis of postoperative infection has become a question that orthopedic surgeons need to pay attention [1–3]. According to statistics, the infection rate of orthopedic surgery is as high as 11.41% and the incision classification of class i, ii, and iii is 1.89%, 7.63%, and 13.08%, respectively [4]. The fluoroquinolone synthetic antibiotic levofloxacin has been widely used in the clinical control of systemic infection due to its advantages of the broad antibacterial spectrum, strong activity, no skin test before use, and no cross-resistance with other antibacterial drugs [5]. At the same time, the adverse reactions of levofloxacin were also more obvious, and unreasonable drug use was an important cause of adverse reactions in patients [6].

Levofloxacin has been widely used in clinical anti-infection treatment because of its wide antibacterial spectrum, high antibacterial activity, and good tissue permeability [7]. However, animal experiments have shown that quinolones can induce irreversible joint damage in young animals, suggesting that quinolones may also have the same toxicity in children, so the application of quinolones in the pediatric field is strictly limited. The drug instructions in the United States and China clearly stipulate that levofloxacin can only be used for the treatment of anthrax in children <18 years old [8]. Levofloxacin has a certain therapeutic value for children with drug-resistant *Mycobacterium tuberculosis* and drug-resistant mycoplasma infection, and relevant clinical studies have also been carried out. Therefore, it is off-label to clarify the occurrence of cartilage damage of levofloxacin.

Levofloxacin is a broad-spectrum fungicide. Its bactericidal mechanism includes acting on dividing cells to inhibit the activity of bacterial DNA rotation, inhibiting the synthesis of RNA and protein, and promoting the phagocytic function of white blood cells. Meanwhile, it also acts on nondividing cells to make them lose viability and thus can cure infection radically. It has the advantages of rapid absorption, high peak concentration, and relatively stable activity. The safety of levofloxacin was improved because of its selective inhibition of topoisomerase ii in bacteria and mammals; the difference between the two was up to 1400 times. Levofloxacin (LVLX) is a new generation of fluoroquinolone drug, which was marketed in 1993. It belongs to the monofouroxacin containing a fluorine group. The structure of levofloxacin is levofloxacin optical isomer, which has stronger antibacterial activity than dextral isomer 8∼128 times is 2 times ofloxacin the clinical dosage of ofloxacin is 1/2. Compared with the first generation of fluoroquinolones, the antibacterial spectrum expanded to Gram-negative cordyceps, Gram-positive chlamydia mycoplasma, and *Legionella* have good antibacterial activity. Good tissue distribution has no cross-infection with other antibacterial drugs, such as drug resistance and other advantages adverse reactions are also greatly reduced, which makes the comprehensive clinical efficacy reach a new level.

Levofloxacin (LVLXDR-3355) is a fluoroquinolone drug developed in Japan in 1986. The active isomer of ofloxacin. It is widely used in clinical practice because of its higher efficacy better tissue distribution lower adverse reactions than ofloxacin. In general, if osteoarthritis is caused by infectious factors, levofloxacin is the drug of choice for treatment, which usually has anti-inflammatory and analgesic effects. However, at present, most osteoarthritis is a disease caused by degenerative changes in the joints, so the use of levofloxacin is not able to achieve a good therapeutic effect. At present, osteoarthritis (OA) is still one of the most common musculoskeletal diseases in the world. OA progresses rapidly, with joint destruction occurring within three to seven years. The pathogenesis of OA is still unclear. Age, infection or inflammation, injury, extra-articular malformation, joint instability, environmental factors, estrogen, excessive weight bearing, obesity, excessive exercise, genetics, diet, and so on the pathogenesis factors. Although infection is not the main factor in the pathogenesis of OA, the discovery of inflammatory cytokines and the current unsatisfactory treatment results inspire us to rethink the role of infection in the pathogenesis and pathogenesis of OA. OA is an inflammatory disease in which a variety of cytokines and inflammatory chemokines are involved in its pathogenesis, among which interleukin plays a major role. At present, it is still controversial whether an infection is the cause of OA, and the role of infection in the occurrence and development of OA is not well understood. Traditional research methods have certain limitations in this respect. With the continuous development of molecular biology technology and means, we can have a deeper understanding of the relationship between infection and OA, thus providing broad prospects for the treatment of OA.

As a common complication of orthopedic patients, the infection has aroused high attention of clinical medical staff, and perioperative prophylactic medication is becoming more and more important. To understand the distribution and drug resistance of common pathogens in bone and joint infection sites of orthopedic patients in our hospital, and to provide an etiological basis for the prevention and treatment of infection [9]. The study showed that there were significant differences in surgical site infection rate among different incisions, underlying diseases, advanced age, long preoperative hospital stay, paralysis and bed rest, use of adrenal glucocorticoids, and implants were risk factors for postoperative infection. At the same time, strengthening the cleaning and disinfection of the ward and the surgical environment, as well as the disinfection and sterilization of instruments and other nondrug prevention strategies are also important links in the control of postoperative infection. In addition, the development of single-tube closed drainage and absorbable artificial bone loaded with antibiotics can also reduce the risk of infection to a certain extent [10].

There are research orifices. It was found that levofloxacin had certain damage to rat, rabbit, and human chondrocytes, but there was a difference in species, rat > rabbit > human. Some studies have found that quinolones can cause reversible damage to the bone joint. Therefore, this study comprehensively collected safety studies and related information on levofloxacin, and evaluated the occurrence of bone and joint adverse events, in order to provide a reference for the off-label use of levofloxacin.

## 2. Materials and Methods

### 2.1. Literature Retrieval

Literature databases: PubMed, Cochrane Library, OVID, EBSCO; Chinese database: CNKI, China Weipu Science and Technology Periodical database, and Wanfang Database. The retrieval time was from January 1993 to 2022 January. Databases under development: WHO clinical trial registration platform (http://apps.whe.int/trialsearch/), American clinical trial registration platform (http://clinieahfials.gov/). Gray literature: proceedings of special conferences, etc., and references of related literature retrospection (Figure 1).

### 2.2. Literature Inclusion Criteria

Inclusion criteria were as follows: (1) subjects were > 18 years old; (2) levofloxacin oral or intravenous infusion, dosage, and course of treatment are not limited; (3) description of any adverse events related to bone and joint, including clinical manifestations and signs (joint swelling, pain, claudication, etc.). Auxiliary examination: X-ray, MRI, and histopathological examination to determine bone and joint changes.

### 2.3. Exclusion Criteria

Exclusion criteria were as follows: (1) the experimental design was nonrandomized controlled literature; (2) for the two literature with the same data, the one published for the first time was regarded; (3) literature that cannot provide valid data for analysis; (4) the second published literature shall be subject to the highest level of the journal; (5) study of combined drug therapy; (6) repeated publications.

### 2.4. Literature Screening

Preliminary screening was conducted through reading articles, and then further screening was conducted after reading abstracts or full texts of literature that might meet the inclusion criteria. If necessary, contact the authors for more research information before making a judgment.

### 2.5. Data Extraction

The main contents include the following: (1) basic information of included literature: author, publication date, country of study implementation, type of study design and sample size, number of lost follow-ups; (2) subjects: age, diagnosis; (3) intervention: drug name, said, dosage and course of treatment, combined medication, and other circumstances; (4) related contents of literature bias risk assessment; (5) outcome indicators. WHO-UMC causality assessment was used to evaluate the association between adverse events and levofloxacin.

### 2.6. Literature Bias Risk Assessment

RCT was conducted in accordance with the risk assessment method of bias recommended in the Cochrane System Evaluator's Manual 5.1.0, which included 6 items randomization, assignment hiding, blinds, the integrity of outcome data, selective reporting of results, and other possible sources of bias, see Figures 2(a) and 2(b)) and Figures 3(a)–3)(d).

### 2.7. Statistical Analysis

For the data of levofloxacin adverse events reported in the literature, OR and 95% CI were used as the effect size for meta-analysis. Descriptive analysis was used when quantitative synthesis was not possible, and *P* < 0.05 was considered statistically significant.

## 3. Result

### 3.1. Literature Retrieval Results and Included Research Characteristics

In this study, PubMed, Cochrane, Web of Knowledge, Embase, CBM, CNKI, CECDB, and CQVIP were searched. A total of relevant literature was retrieved during the initial screening. Repeated publications and RCTs were excluded by reading titles and abstracts, and 19 literature were left. 19 full papers were reviewed, different reports of the same clinical study and literature inconsistent with the content of this study were excluded, and references of relevant literature were searched to prevent literature omission. Finally, a total of 12 RCTs were included in the study [11–24]. All the retrieval and screening processes were completed by two evaluators independently, and any different opinions were unified through internal discussion (Table 1).

### 3.2. Incidence of Fever

Among the 14 RCTs' literature included in the incidence of fever, a heterogeneity test was carried out and it was found that the heterogeneity of the selected studies was small, so a meta-analysis with fixed models could be performed. The results of the meta-analysis showed that the rhombus plot and vertical line no intersected in the forest map of incidence of fever for 4 included literature, so there was a statistical difference in the comparison of the incidence of fever between the experimental group and the control group (OR = 2.29, 95% CI (1.75, 2.98), *P* < 0.00001, *I*^2^ = 0%, *Z* = 6.11) (Figure 4).

### 3.3. Elevated White Blood Cell Count

Among the 14 RCTs' literature included in elevated white blood cell count, a heterogeneity test was carried out and it was found that the heterogeneity of the selected studies was small, so a meta-analysis with fixed models could be performed. The results of the meta-analysis showed that the rhombus plot and vertical line no intersected in the forest map of elevated white blood cell count for 4 included literature, so there was a statistical difference in the comparison of elevated white blood cell count between the experimental group and the control group (OR = 1.82, 95% CI (1.31,2.52), *P*=0.0003, *I*^2^ = 0%, *Z* = 3.60) (Figure 5).

### 3.4. Incidence of Wound Infection

Among the 14 RCTs' literature included in the incidence of wound infection, a heterogeneity test was carried out and it was found that the heterogeneity of the selected studies was small, so a meta-analysis with fixed models could be performed. The results of the meta-analysis showed that the rhombus plot and vertical line no intersected in the forest map of incidence of wound infection for 4 included literature, so there was a statistical difference in the comparison of the incidence of wound infection between the experimental group and the control group (OR = 2.11, 95% CI (1.54,2.90), *P* < 0.00001, *I*^2^ = 0%, *Z* = 4.64) (Figure 6).

### 3.5. Adverse Drug Reaction

Among the 14 RCTs' literature included in adverse drug reactions, a heterogeneity test was carried out and it was found that the heterogeneity of the selected studies was small, so a meta-analysis with fixed models could be performed. The results of the meta-analysis showed that the rhombus plot and vertical line no intersected in the forest map of adverse drug reactions for 4 included literature, so there was a statistical difference in the comparison of adverse drug reactions between the experimental group and the control group (OR = 1.82, 95% CI (1.21,2.74), *P*=0.004, *I*^2^ = 0%, *Z* = 2.86) (Figure 7).

## 4. Discussion

The efficacy of perioperative antibiotics in preventing surgical infection has been widely verified in clinics [25]. Levofloxacin has been widely used in the prevention of postoperative infection due to its wide antibacterial spectrum, strong antibacterial activity, and low drug resistance rate, as well as its unique pharmacokinetic characteristics, such as 5.8 h half-life, high tissue concentration, and no skin test [26]. However, in the clinical application of levofloxacin as a broad-spectrum antibiotic, adverse drug reactions also occur from time to time. In addition to the influence of individual differences and other objective factors, in order to effectively reduce the incidence of ADR, ensure the health of patients and minimize the pain of patients, clinicians need to make a comprehensive analysis of the clinical data of patients [27–30].

Surgical site infection is one of the most common postoperative complications, surgical site infection, particularly surgical site infection of the incision, the most direct impact is delayed healing of the incision, appear even incision split, more serious may lead to the surgical site physical disability and corresponding organ dysfunction or failure, there is also a cause of deaths; therefore, we must pay attention to the occurrence of surgical site infection complications, and adopt effective prevention and treatment measures. Surgical site infection complications occurred more influencing factors, such as the surface of the operating room environment and air quality, skin disinfection of operation, quality of equipment, the performer such as hand hygiene can cause late complications, surgical site infection in patients with surgical site infection and disease occurrence is necessary to real-time monitoring, and adopt specific measures to prevent complications of infection, Through the implementation of “whole-process quality management” measures to reduce the incidence of surgical site infection complications. In order to better understand the incidence of surgical site infection in patients with bone and joint surgery, and to obtain effective prevention and treatment measures for complications. The overall results showed that the complications of bone and joint surgery site infection were mainly in type I incisions, accounting for 83.33% of all infected patients. The results also showed that there was a certain correlation between surgical risk index and the incidence of surgical site infection complications, that is, the higher the surgical risk index, the higher the incidence of surgical site infection complications; It is suggested that the prevention of infection complications should be prepared before determining the risk index of surgery and performing surgery, so as to reduce the probability of complications of surgical site infection. We also see the importance of implementing whole-process quality management. In terms of perioperative medication, this study believes that the proportion of patients taking drugs should be reduced and targeted medication should be increased. Moreover, antibacterial drugs of the first generation cephalosporin should be the main drug, and antibacterial drugs of the third generation cephalosporin should not be directly used.

Over 60 years old in patients receiving levofloxacin there was a higher incidence of adverse reactions to prevent infection treatment mainly includes: the main reasons for elderly patients with viscera function decline, easily complicated by a variety of disease, and levofloxacin by kidney metabolism, effects on kidney burden, clinical applications in the old people should take into consideration the reduction and regular monitoring of kidney function [31]. In addition, from the animal experiments on quinolone antibiotics, it was found that young animals taking quinolone antibiotics would produce cartilage damage to joint tissue, so children, pregnant and lactating women should be forbidden levofloxacin [32–35]. At the same time, because levofloxacin belongs to quinolones antibiotic effect, from this group of cases cure effect and ADRs of reaction after taking levofloxacin, static drop 1- or 2-times daily fee sand star of left oxygen drugs for prevention of postoperative infection, there was no significant difference, and oxygen cost effect of medication to reduce the incidence of ADR is safer and more effective [36–39].

To sum up, levofloxacin should be paid attention to the following points in preventing infection after bone joint and internal fixation: (1) when prescribing levofloxacin, the patient's physical condition should be consulted in detail. If the patient is allergic, it should be avoided as far as possible; (2) the storage temperature of levofloxacin and other drugs should be controlled within 20°C and stored away from light to prevent improper storage and degradation of drugs, reduce pharmacological effect and cause adverse reactions; (3) patients should eat before infusion, to avoid drug reaction to aggravate the stimulation of empty abdomen, so that gastrointestinal discomfort magnify; (4) pay attention to keep the infusion speed slow, 100 ml infusion time is not less than 1 h; (5) pay attention to the patients with liver and kidney function decline, especially the elderly patients, for the weak patients with levofloxacin in vivo clearance rate reduced, the half-life prolonged, in order to prevent drug accumulation caused toxicity, doctors must reduce the drug dosage; (6) levofloxacin can pass through the blood-brain barrier, into the brain tissue and may cause central nervous system reaction, for patients with cerebrovascular disease, epilepsy or family history of mental illness and other basic diseases of the central nervous system, should pay attention to control or prohibit the use. As a common complication of orthopedic patients, the infection has aroused high attention of clinical medical staff, and perioperative prophylactic medication is becoming more and more important. In order to understand the distribution and drug resistance of common pathogens in bone and joint infection sites of orthopedic patients, and to provide an etiological basis for the prevention and treatment of infection. The risk factors for postoperative infection were underlying diseases, advanced age, long hospital stay, paralyzed bed, use of adrenal glucocorticoids, and implants. At the same time, strengthening the cleaning and disinfection of the ward and surgical environment, as well as the disinfection and sterilization of instruments and other nondrug prevention strategies are also important links in the control of postoperative infection. In addition, single-tube closed drainage and absorbable artificial bone technologies can also reduce the risk of infection to a certain extent.

Available evidence shows that the incidence of osteoarticular adverse events with levofloxacin is low and most of them are resolved during follow-up. It can provide a basis for the off-label use of levofloxacin after fully evaluating the risks and benefits.

## Figures and Tables

**Figure 1:** Flow chart of the literature screening.

**Figure 2:** Literature quality evaluation chart. (a) Risk of bias graph. (b) Risk of bias summary.

**Figure 3:** a-d: Funnel plot of literature publication bias.

**Figure 4:** Meta-analysis of incidence of fever between two groups.

**Figure 5:** Meta-analysis of elevated white blood cell count between two groups.

**Figure 6:** Meta-analysis of incidence of wound infection between two groups.

**Figure 7:** Meta-analysis of adverse drug reaction between two groups.

**Table 1:** Basic clinical features of 14 literature were included in our study.

Study	Age	Gender (Male)	(%) Experimental group (N)	Control group (N)	NOS score
Meléndez-Carmona MÁ 2019	53.71 ± 12.2	41.25	42/65	30/65	8
Asseray N 2016	55.65 ± 13.4	69.12	160/260	100/260	7
Tornero E 2016	63.12 ± 14.5	45.72	78/143	54/143	8
Lora-Tamayo J 2016	67.15 ± 14.5	44.12	100/175	75/100	8
Bernard A 2015	52.85 ± 8.4	51.89	20/34	14/34	8
Yoda T 2000	64.36 ± 10.2	63.45	24/44	20/44	7
Qiao J 2022	62.62 ± 12.2	78.10	30/50	20/50	9
Gergs U 2018	62.61 ± 13.0	48.75	26/42	16/42	9
Canouï E 2022	57.25 ± 14.5	59.23	62/102	40/102	7
Eloy G 2020	66.22 ± 15.2	56.22	32/59	27/59	8
Ferreira M 2017	61.35 ± 8.1	53.16	25/45	20/45	8
Matos AC 2015(1)	57.25 ± 16.0	66.34	22/35	18/35	8
Matos AC 2015(2)	58.51 ± 8.6	48.34	48/67	35/67	9
Wang Q 2017	66.34 ± 6.5	53.12	55/66	42/66	9

## Data Availability

The data used to support this study are available from the corresponding author upon request.
